The article "Research and Implementation of Distributed Computing Management System for College Students' Sports Health Based on Integrated Regional Collaborative Medical Care" was retracted in 2023. Reasons: signs of a paper mill; suspected computer-generated content; unreliable results or conclusions; lack of ethics approval or compliance.

# Research and Implementation of Distributed Computing Management System for College Students' Sports Health Based on Integrated Regional Collaborative Medical Care

**DOI:** 10.1155/2022/9306200

**Published:** 2022-05-18

**Authors:** Mian Wang, Lijuan Li

**Affiliations:** ^1^School of Science and Technology, Nanchang University, Jiangxi 330006, China; ^2^Sports Institute, Nanchang University, Jiangxi 330006, China

## Abstract

This paper constructs and applies a university student sports health management system through the theory of integrated regional collaborative medical care and distributed computing technology. Firstly, it analyzes the current situation and problems of cross-regional medical care, the root causes, and the corresponding business scenarios, reflecting the development trend of cross-regional medical care, in the light of the current practical needs of cross-regional medical care. In response to the strong demand for cross-regional medical care, this paper gives the overall design of the distributed computing system, for the deployment and architecture of the cross-regional platform; the registration of cross-regional patients, regional platforms, and health events and documents; and data exchange, service integration, and process integration, etc. The corresponding design is given. The research was conducted on several medical institutions to refine the functional requirements for the construction of the regional collaborative medical platform, and the requirements were analyzed to present the research results of the collaborative medical project. Based on this, requirements were made for the preparation of the project construction data center and medical institutions, and the remote consultation and two-way referral modules of the distributed collaborative medical platform were designed, which are processed and analyzed through a system composed of multiple servers. The results are returned to the user, and the design results were tested for functionality, compatibility, security, and other usability tests. The necessity and feasibility of the college physical health test data platform were analyzed. Students have various needs for physical test data management, the necessity of designing the college physical health test data platform, and the feasibility of the college physical health test data platform in terms of technical means, theoretical basis, and social environment.

## 1. Introduction

Health management is to determine the health status of users through comprehensive monitoring and analysis of health behaviors and to provide health consultation and intervention services to users [1]. Its purpose is to mobilize the initiative of individuals, encourage people from all occupations to contribute to health management services, and make full use of available resources to improve health management effects. In carrying out sports health management services, the same step-by-step requirements of information management, health assessment, health intervention, supervision, and feedback of health management are followed, with the difference that the sports health management service system focuses on health intervention utilizing sports. As a transitional period between school education and social practice, the most important task in this period is to enhance the awareness of sports health management among college students, to promote them to develop sports habits and stimulate their interest in sports, and then to realize the purpose of lifelong sports [2]. At the same time, it is also required for students that young people should be proficient in more than one sporting skill, ensure at least one hour of physical exercise every day, and meet the standard of a physical fitness test for college students.

The article "Research and Implementation of Distributed Computing Management System for College Students' Sports Health Based on Integrated Regional Collaborative Medical Care" was retracted in 2023. Reasons: signs of a paper mill; suspected computer-generated content; unreliable results or conclusions; lack of ethics approval or compliance.

Nonoperating government investment projects, as a kind of public utility projects not for profit, are different from operating government investment projects, and their public and social nature is particularly important in the process of project construction, so the planning and decision-making process of nonoperating government investment projects should be based on facts and scientific decision-making means, and strive to maximize the satisfaction of public demand [3]. However, due to the complexity of nonoperating government investment projects, it is difficult to make a fair, scientific, and efficient decision-making plan by relying on the government's power alone, which also leads to many decision-making errors in its project decision-making and causes a large amount of waste of national resources [4–9]. As a kind of nonoperating government investment project, it is difficult to ask consumers to remain rational because it involves the medical industry and involves life. Our medical system model is a state-owned private system model, where the government takes the lead in setting prices on the one hand, while still being able to operate on the other, and this medical system model has led to an imbalance in our medical resources [10–12]. The most obvious one is that the quality of medical care varies greatly between the top tertiary hospitals and the various primary hospitals in China, while the prices are very different, which inevitably leads to an influx of patients, regardless of the severity of their illness, to the high-level large hospitals in the hope of receiving the best quality medical care.

The article "Research and Implementation of Distributed Computing Management System for College Students' Sports Health Based on Integrated Regional Collaborative Medical Care" was retracted in 2023. Reasons: signs of a paper mill; suspected computer-generated content; unreliable results or conclusions; lack of ethics approval or compliance.

The main purpose of this study is to improve health and maintain health status. The goal is to enhance health management awareness, develop exercise habits, and stimulate interest in exercise [13–18]. With the help of smart devices such as the Internet and cell phones, to achieve the goals of health information collection, health status assessment, development of health thousand preplanning, and monitoring and implementation [19], the health interventions are mainly to develop and implement exercise prescriptions and recommended exercise programs to help students achieve the goal of improving health and maintaining health status by improving health risk factors, strengthening the sense of accomplishment in exercise participation, and increasing the number and duration of exercise participation, to achieve the ultimate goal of enhancing exercise health management awareness, cultivating exercise habits, and stimulating exercise interest [20–25].

A regional medical center project is a kind of nonoperating government investment project, which is a kind of public facility investment project with taxpayers' money. In the process of investment decision research on the regional medical center projects, some key points in the investment decision of nonoperating government investment projects can also be referred to [26–28]. This single organization coordinates and distributes tasks and controls costs through the network. It is specialized and core, and it is beneficial for people to receive the most valuable services in the most suitable locations. In the research of nonoperating government investment projects, the DEA-Tobit investment decision model is proposed by improving the Tobit method and evaluating the overall efficiency of the government investment project group and branch project efficiency from the micro perspective, highlighting the key position of capital and social benefits in the index system in the evaluation process, and prioritizing the efficiency evaluation impact factor indexes, which can help managers to analyze the problems arising in the project decision-making [29–31]. A public participation performance index system is constructed to study the effect of public participation in government investment projects, and then, the practicality of this public participation index system is verified through actual cases [31–33]. The investment effects of government industrial funds are studied, and some policy suggestions are provided for the improvement of institutional norms and the utility of government industrial fund investment from the design of the relevant system of government industrial funds.

A group decision-making method based on regret theory is proposed to make decisions on uncertain linguistic evaluation values, and the regret psychology of decision-makers is considered in the decision-making model, and the model is verified through practical cases [34–36]. Taking the new product development decision as to the research object, the group decision process is integrated into the fuzzy best-best method, and a decision model for new product idea decision is constructed by a combination decision method, which contributes to the field of new product development. Based on the classical full method, a group decision model based on interval intuition fuzzy number is constructed to study the quantitative evaluation problem in social networks, and the limitations of subjective empowerment are well solved in the decision process, and finally, the practicality of the model is verified by the dynamic evaluation case of Sine Weibo users' influence [37].

The article "Research and Implementation of Distributed Computing Management System for College Students' Sports Health Based on Integrated Regional Collaborative Medical Care" was retracted in 2023. Reasons: signs of a paper mill; suspected computer-generated content; unreliable results or conclusions; lack of ethics approval or compliance.

Practical needs have motivated the development of health research. The irregularity of people's lives, the influence of work, the influence of living environment, or the influence of bad habits in modern society have prompted people to develop various physical and psychological disease problems, with a wide variety of diseases and a wide range of incidence rates increasing year by year. To cope with the emergence of diseases and to meet the needs of work and life, health management along with people's physical health improvement needs to follow the trend [38]. Nonpharmacological management of human physical health does not require medication, does not have side effects on the human body under the premise of science, can be implemented in any location, and has the effect of improving the overall health of the human body, which is a method of improving physical health more adapted to modern lifestyles. After studying and analyzing the above literature on medical centers and government investment, it can be found that at this stage, most of the articles on regional medical center research focus on site selection, medical center management models, and medical services, and most of the literature on government investment focuses on project supervision and use of project funds. The focus of the literature on the location of medical centers has been on the optimization of path algorithms and decision-making methods, with little consideration given to the synergistic effect of the development of regional medical centers on the surrounding radiation areas.

## 2. Methods

### 2.1. Design

The essential feature of a collaborative network is to establish strategic synergistic relationships among subjects through the collaborative use of resources, systems, and technologies to achieve the common goals of each subject. Division of labor, differentiation, and integration are the three basic units of cooperation, which together drive the evolution of an organization from a single entity to an organizational community. In this process, the organizational technology keeps advancing, the cognition of cooperation concept tends to be consistent among all subjects, and the differentiation and integration among organizational clusters become deeper, gradually forming a three-dimensional network based on clusters [39]. The degree of organization of each industry in a country or society is closely related to the scale and complexity of the network. The formation of a regional medical collaborative network can promote consensus among medical institutions within the network, improve the efficiency of communication and coordination, and allocate resources [40]. However, regional healthcare services also require the creation of various organizational forms due to the varying capabilities of healthcare institutions at all levels and the different consumer preferences, payment capacity, and willingness.

The article "Research and Implementation of Distributed Computing Management System for College Students' Sports Health Based on Integrated Regional Collaborative Medical Care" was retracted in 2023. Reasons: signs of a paper mill; suspected computer-generated content; unreliable results or conclusions; lack of ethics approval or compliance.

Operating and management rights are unified, with the autonomy of operation, the ability to flexibly adjust the direction and mode of operation according to changes in service demand and policy environment, and the corresponding responsibility for the operation [41]. The most important management rights mainly include the right to make business decisions and the right to allocate resources. The organizational approach and management are diverse. The organizational approach is mainly a strategic partnership based on the social public nature of medical institutions and medical services and common goals, and its management is mainly characterized by the principles of public management, such as representativeness, transparency of procedures, and reflectiveness of needs [42]. The single organization becomes a cost center within the network, controlling costs by keeping the population healthy and providing appropriate care, and the network needs to work to optimize organizational operational efficiency and redesign clinical processes so that people can receive the best value in the most appropriate location. This single organization coordinates and distributes tasks and controls costs through a network that is specialized and centralized so that people can receive the best value in the most appropriate location.

Management cooperation is an all-around cooperation of organizational goals, structure and organization, production and operation, technology and methods, supervision and control, and culture of each subject, which requires the best effect of integrating and using resources [43]. The core concept is to reconstruct and integrate, that is, to reconstruct organizational methods, rules, and procedures to achieve overall goals, and to comprehensively allocate and coordinate the use of resources to achieve the best results. Management cooperation is to improve the quality and level of services and balance the number of services in an integrated manner by strengthening coordination and management and promoting the rational use of resources to output the best results. It builds a rational, efficient, and risk-controlled medical access procedure and a process-oriented quality management system, resource sharing, and collaborative call.

The article "Research and Implementation of Distributed Computing Management System for College Students' Sports Health Based on Integrated Regional Collaborative Medical Care" was retracted in 2023. Reasons: signs of a paper mill; suspected computer-generated content; unreliable results or conclusions; lack of ethics approval or compliance.

The cross-regional medical sharing and collaboration system provide common basic functions for cross-regional medical information sharing, including cross-regional unique patient identification, regional information platform registration, medical institution registration, event registration, document registration, indexing services, business collaboration-oriented distributed medical resource management, off-site treatment information sorting services, and cross-regional business process management services. The overall architecture is shown in Figure 1.

The business of cross-regional medical sharing and collaboration system is complex and involves various aspects of data of cross-regional patients seeking medical treatment in different places, such as electronic medical records with unstructured characteristics and medical images with large quantity and capacity, and different data types have different storage requirements [44].

The so-called hybrid storage is compatible with both centralized and distributed storage methods. The centralized storage is to store the data within the scope of health records in a unified data center, which mainly focuses on document data; the distributed storage is to store the content of large files and the content of health records that cannot be structured and is called very infrequently in the data center, considering the storage capacity and network bandwidth, and the data center indexes the location information of these files [45]. When the demand side makes a call, it searches for the file location through the index of the data center, then loads it into the cross-regional medical collaboration system, and then provides it to the content demand side for use. This storage method is recommended for large-capacity files such as medical image data and voice data.

In the primary data center, we deploy clinical collaborative application server, collaborative supervision server, image PACS server, image browsing server, image report server, audio and video server, distance education server, collaborative interface server, collaborative database server, collaborative resource storage server, data, and image storage; the same city backup data center realizes real-time synchronous mirroring of virtual machines and once the hardware or application of the primary. Different data types have different storage requirements. Here, we consider using a hybrid storage method to store data. Once the hardware or application of the primary data center has a problem, the hardware or application of the backup data center can be switched instantly.

The article "Research and Implementation of Distributed Computing Management System for College Students' Sports Health Based on Integrated Regional Collaborative Medical Care" was retracted in 2023. Reasons: signs of a paper mill; suspected computer-generated content; unreliable results or conclusions; lack of ethics approval or compliance.

### 2.2. Functions

The physical education department is the core of the physical health management system, responsible for teaching students' health theoretical knowledge, as well as setting up students' sports programs and arranging extracurricular activities. Physical education teachers formulate specialized teaching programs based on physical and mental health development and make timely adjustments according to students' physical fitness level and skill learning proficiency during curriculum development to improve students' awareness of the importance of sports and their exercise [46]. Sports assist college students to cultivate good exercise habits and help them to form a healthy lifestyle.

The physical fitness test data platform for college students does not appear out of thin air but is based on the real needs of real-life and has the necessary theoretical design and construction. There are three specific needs of the physical health test data platform for college students [47]. The first one is user requirements. The main users of the physical fitness test data platform for college students are students, physical education teachers, and some school sports managers, so it is necessary to design and develop the corresponding functions of the physical fitness test data platform for college students according to the needs of each part of users. At the same time, because the universities are in different regions, the management systems of the universities themselves are different, and the main body of students in the universities is also different; it is necessary to meet the needs of users in the actual design according to the situation.

Students are the main subjects in student sports work in universities, and the purpose of school sports work is also to enhance students' physical fitness, as shown in Figure 2. Therefore, it is necessary to manage students' physical health based on physical fitness test data [48]. By distributing questionnaires to students in six schools in Changchun, students' demand for physical health management based on physical health test data is investigated as shown in the following figure: students who think it is very necessary to manage physical health test data account for about 35% of the number of college students surveyed, those who think it is necessary to manage physical health account for about 45% of the number of students surveyed, and those who think it is not necessary to account for about 8% of the number of students surveyed. Those who think it is not necessary are about 8% of the surveyed students, and those who are indifferent are about 17%. This shows that students in six schools in Changchun have a strong demand for physical health management based on physical health test data, which shows that students in universities generally have a positive attitude toward physical health management.

The article "Research and Implementation of Distributed Computing Management System for College Students' Sports Health Based on Integrated Regional Collaborative Medical Care" was retracted in 2023. Reasons: signs of a paper mill; suspected computer-generated content; unreliable results or conclusions; lack of ethics approval or compliance.

Taking students as the main body and taking students' needs as the guide are the starting point of this study in the theoretical design of the physical health test data platform for college students; therefore, it is the basic work to understand the students' demands for the data platform. Through the survey of students in six schools in Changchun, the functional demands of college students on the data platform of college students' physical fitness tests are shown below [49]. The survey found that about 59% of students want to get exercise skill instruction; about 67% want to get targeted exercise prescription design; about 72% want to get physical education course resources; about 58% want to establish physical health records; about 71% want the platform to provide physical quality evaluation; about 21% want the platform to provide exercise theory knowledge education. About 9% of students have other requirements, as shown in Figure 3.

### 2.3. Modules

For the establishment of functional indicators of physical fitness test data platform for college students, this study adopts the following ideas to establish indicators: collecting functional indicators ⟶ screening functional indicators ⟶ determining functional indicators ⟶ forming a framework system. At present, by reviewing the literature, we can know that there are already many functional indicators on the management of physical health of college students, the system of student physical fitness monitoring, and the management of student physical test data. Therefore, this study collects the indicators established by previous studies, considers the current practical needs of college students and teachers, screens the functional indicators of the college student physical fitness test data platform, and finally constitutes the college student. Finally, the framework system of the data platform of college student physical fitness test is formed.

The article "Research and Implementation of Distributed Computing Management System for College Students' Sports Health Based on Integrated Regional Collaborative Medical Care" was retracted in 2023. Reasons: signs of a paper mill; suspected computer-generated content; unreliable results or conclusions; lack of ethics approval or compliance.

Finally, three primary indicators of the functional module of the college student physical health test data platform are formulated, and two secondary indicators and five tertiary indicators are divided under the functional module of student physical health data monitoring. There are 5 secondary functional indicators and 13 tertiary functional indicators under the student physical health intervention function module and 4 secondary functional indicators and 13 tertiary functional indicators under the school sports resources and information function module, as shown in Table 1.

The modern concept of health does not mean simply the absence of disease in the body; as people's understanding of health becomes deeper and deeper, the concept of health has moved from one-dimensional to multiple dimensions in terms of physiological, psychological, and social adaptability. To monitor the physical health of students in colleges and universities, it is inevitable to realize the close association of sports department, school hospital department, and school psychological guidance center to realize the all-round monitoring of students, and the relationship structure of the three departments is shown in the figure below. Therefore, the basic data collection of students should be based on students' physical health test data, covering students' medical physical examination data and psychological assessment data. Students' basic data can be collected by manual entry or by importing Excel tables.

Students' behavioral data is the feedback to the school's physical education work, which is the invisible data behind the students' basic data. The students' behavioral data can be collected and analyzed to better realize the physical health monitoring of students. There are two main categories of behavioral data collection: one is data collection during physical education courses, and the other is information collected from after-school physical education activities [50]. The data center indexes and stores the location information of these files and does not store their actual data. When the demander makes a call, it finds its file location through the data center index, and then loads it into the cross-regional medical collaboration system, and then provides it to the content demander for use. The collection can be done through questionnaires and interviews with students. With the maturity and popularity of fitness devices, such as sports bracelets and sports watches, it is possible to monitor the heart rate data in real-time during physical education classes and after-school sports activities and transmit them to the management platform in time for targeted analysis of exercise intensity. In addition, the relevant sports monitoring software in cell phones is becoming increasingly perfect, such as WeChat Sports and keep, which can be used to transfer the whole exercise data of college students to the platform for analysis in time.

The article "Research and Implementation of Distributed Computing Management System for College Students' Sports Health Based on Integrated Regional Collaborative Medical Care" was retracted in 2023. Reasons: signs of a paper mill; suspected computer-generated content; unreliable results or conclusions; lack of ethics approval or compliance.

The second part is the function of sports prescription, which mainly intervenes in students' after-school sports activities, and this function is realized mainly by establishing the expert system of sports prescription. The expert system is an intelligent computer program built into the physical health test data platform of college students, which writes the experience and various theoretical knowledge of experts in the field of exercise prescription and simulates the way of thinking of experts in the field of exercise prescription to design a scientific and reasonable exercise prescription for each student's specific situation. By analyzing the data of the student's physical fitness test results, the expert system calculates the exercise intensity that the student can adapt to; quantifies the specific exercise time, frequency, and load size; and designs a weekly exercise prescription based on the student's choice of sports and personal interests in physical education classes. The exercise prescription will be sent back to the teacher, who will decide whether it is reasonable and implemented. After the implementation, students are required to clock in and out to monitor the students. Finally, students evaluated the exercise prescription according to their feelings.

## 3. Results

The qualitative indexes in this paper involve four major aspects: economic, social, environmental, and regional synergistic development, because of their wide scope and many subject areas. The expert evaluation method cannot give detailed evaluation values for such complex projects but can only evaluate and score the evaluation indexes with fuzzy language values through the experience and knowledge of experts in each field. The overall process of qualitative index evaluation is to have a team of experts discusses and analyze the alternatives; then, the experts score the linguistic values and finally convert the linguistic values into interval intuitionistic fuzzy numbers.

### 3.1. Scoring

Firstly, the expert team scored the indicators of the regional medical center project index system using linguistic values, and there are seven types of evaluation linguistic values set in this paper: very high, high, average high, average, -average low, low, and very low. For example, when experts are required to score the construction cost index of the alternative, after the analysis of expert A's expertise and experience, the construction cost of the site is considered high, and the affiliation degree of the construction cost index is “high”; then, the evaluation result of expert as for this index can be expressed as ([0.7, 0.8]. [0.1, 0.2]). Intuitive fuzzy number conversion between zones is shown in Table 2.

The article "Research and Implementation of Distributed Computing Management System for College Students' Sports Health Based on Integrated Regional Collaborative Medical Care" was retracted in 2023. Reasons: signs of a paper mill; suspected computer-generated content; unreliable results or conclusions; lack of ethics approval or compliance.

For the quantitative indicators in the investment decision project of the regional medical center of the economic community, they are generally obtained through on-site measurements. The four quantitative indicators can be obtained from the government statistical yearbook and the government development bulletin, and the engineering pollution purification power can be obtained by calculation. To facilitate the latter calculation, after obtaining these quantitative indicators, it is necessary to convert them into interval intuitionistic fuzzy numbers uniformly and carry out normalization to eliminate the influence of the dimension.

As the concept of regional synergistic development of urban agglomerations continues to grow, the members of the project decision-making expert committee hope to make the construction of the project drive the economic development of all cities within the region and the development of the medical industry as much as possible, while satisfying the basic engineering of the project.

The quantitative indicators in this paper are mainly 5, all of which are benefit-based quantitative indicators. The specific data of transportation resources and medical resources used in this paper are obtained through specific information, which can be found in national statistical yearbooks and regional government development reports. The construction pollution purification power can be calculated through calculation formulas and related research literature. The population of the radiation area is found through comprehensive national yearbook information. The number of cities within the radiation area is found through map data of various places. After the quantitative data collected, the quantitative data are de-quantified and converted into interval intuition fuzzy numbers, and the evaluation value of the converted quantitative indicators is shown in Figure 4.

Regional collaborative medical service is centered on regional medical data and explores the business process and digital guarantee system of collaborative service utilizing medical information exchange, sharing, and interoperability to enhance the convenience of regionalized means of medical consultation. Large general hospitals provide remote collaborative medical services based on regional medical information integration and sharing directly to other medical institutions at all levels, thus realizing regional radiation and point-to-point collaboration, especially for the immediate disposal of emergency cases.

The article "Research and Implementation of Distributed Computing Management System for College Students' Sports Health Based on Integrated Regional Collaborative Medical Care" was retracted in 2023. Reasons: signs of a paper mill; suspected computer-generated content; unreliable results or conclusions; lack of ethics approval or compliance.

### 3.2. Performance

Axure BP is a professional rapid prototyping tool developed by Axure in the U.S. It has a simple interface and modular functional components, which can design products with good interaction effects. It has a simple interface and modular functional components, which can design a product prototype with a good interaction effect, express the product content clearly, and is easy to postproduction and maintenance. In this paper, the interface and interaction design of the computer-based student client of the university physical fitness test data platform are carried out by the Axure RP software.

At present, the time for college students to participate in sports is seriously compressed, the number of participants in extracurricular sports activities is relatively small, and the participation items are concentrated. In the current investigation and research on the participation of extracurricular sports activities, although the current situation of college students' participation in sports has been analyzed and corresponding suggestions have been put forward, there is not much involvement in practice, and there is a lack of research on practical measures.

The subhealthy state is prevalent. The subhealth state is mainly reflected in three aspects: physical health, mental health, and social health. As shown in Figure 5, 46.3% of students have good physical health, 83.3% have good mental health, 76.4% have good social health, and only 5.5% have no sports-related injuries or illnesses. Combined with the data of this survey, it is easy to find that a large proportion of students are in a subhealthy state, and sports injuries and illnesses are common. Prevention and management of sports-related injuries are necessary.

In the survey of students who failed the physical test, 71.8% of the students were aware of health management but did not apply it, and 17.2% did not understand the concept of sports health management or even did not know it at all. Not knowing and not using exercise health management is an important reason for the decline of the physical health level of college students. Therefore, establishing a convenient and scientific exercise management system and encouraging students to take the initiative in health management are a real problem that needs to be urgently solved by the current research. The school reasonably arranges students' physical fitness test work, strengthens the supervision of students' physical fitness test, and ensures effective physical performance. The students' physical fitness test scores are archived, and the students' physical health status is analyzed and graded.

The article "Research and Implementation of Distributed Computing Management System for College Students' Sports Health Based on Integrated Regional Collaborative Medical Care" was retracted in 2023. Reasons: signs of a paper mill; suspected computer-generated content; unreliable results or conclusions; lack of ethics approval or compliance.

Understanding what each health indicator represents is a prerequisite for self-exercise health management. However, in the whole survey, 34.9% of the students could not judge their health through the health test results, and only 31.5% of the students could improve their physical health according to the physical test results. The reasons for this problem include the lack of basic knowledge of health management among college students and the lack of a convenient exercise health management system for students to use in their daily life. The development and design of an online exercise and health management service platform can solve the problem of lack of health management knowledge among college students.

Participation in sports and health management can effectively maintain physical health and enhance physical fitness, and it can be said that interest in sports is the source of motivation for sports health management and participation in sports. However, there is a general lack of exercise interest among college students, as shown in Table 3. 30% of the students who failed the physical test did not have an interest in sports; 25.4% of all the sampled students did not have exercise interest; 8.9% of the students who had exercise interest did not know that their favorite sports would be helpful to their physical health. For students without exercise interest, 99.0% of them would accept the recommended exercise program. Therefore, there is a greater demand for students to obtain scientifically recommended exercise programs.

The health management system is more far-reaching, with the concept of lifelong sports running throughout the health management system. Health self-management is the basis for users to develop health management habits, and the exercise health management system designed in this paper provides practical tools for college students to carry out health self-management. The health management service system can update the content of exercise prescription according to the current health status and behavior of users, effectively encourage users to actively participate in sports, increase participation in sports, and realize the transformation from passive exercise to active exercise. In the process of participating in sports, we can improve the subhealth status and stimulate the interest in sports.

Option recommendation is more personalized, and current research on exercise option recommendation systems focuses on two aspects: recommendation of choosing special physical education classes and recommendation of choosing exercise programs. About 72% of students hope to get physical education resources; about 58% of students hope to establish physical health records; about 71% of students hope that the platform provides physical fitness evaluation; about 21% of students hope that the platform provides sports theoretical knowledge education. The former is more influenced by external factors such as school curriculum and teachers, but essentially, it also recommends specific sports for users. The latter research is more focused on analyzing users' characteristics and similarities among users, which requires a certain user base and neglects the relationship between sports items. In this paper, by analyzing the characteristics of different item groups, we clarify the relationship between sports items, then match the sports items of different categories according to the users' health needs, and finally select suitable sports items among the group categories and recommend them to the users by combining the influence of the actual situation around the users.

The article "Research and Implementation of Distributed Computing Management System for College Students' Sports Health Based on Integrated Regional Collaborative Medical Care" was retracted in 2023. Reasons: signs of a paper mill; suspected computer-generated content; unreliable results or conclusions; lack of ethics approval or compliance.

## 4. Discussion

In this paper, we analyzed in detail the current situation of the construction and development of regional medical consortia from four dimensions. It was found that there are multiple problems such as loose alliance among the members of the medical consortium in Yantian Prefecture, unsound management mechanism within the medical consortium, insufficient continuity of medical services, and low sharing of medical information resources. The necessity and feasibility of the physical health test data platform in colleges and universities were analyzed. Students have various needs for physical health test data management, the necessity of designing the physical health test data platform in colleges and universities, and the feasibility of the physical health test data platform in colleges and universities in terms of technical means, theoretical basis, and social environment. The theoretical design was carried out for the physical health test data platform for college students, and the functional modules of the platform were screened and designed: student physical health data monitoring, physical health intervention, school sports resources, and information. In the actual operation of the physical health test data platform for college students, corresponding systems are formulated and strictly implemented; the normal operation of the platform is guaranteed by regular maintenance of the later stage of the physical health test data platform for college students.

## Figures and Tables

**Figure 1:** Architecture of medical sharing and collaboration system.

**Figure 2:** Students' demand for physical health management based on physical health test data.

The article "Research and Implementation of Distributed Computing Management System for College Students' Sports Health Based on Integrated Regional Collaborative Medical Care" was retracted in 2023. Reasons: signs of a paper mill; suspected computer-generated content; unreliable results or conclusions; lack of ethics approval or compliance.

**Figure 3:** Students' demands for the functions of the physical fitness test data platform for college students.

**Figure 4:** Evaluation value.

**Figure 5:** Health status.

**Table 1:** Functional module screening table of the physical health test data platform for students in colleges and universities.

First-level indicator	Secondary indicators	Three-level indicator
Physical education program resources and information	Basic data	Physical test data
		Medical examination data
		Psychometric data
		Physical education activity data
	Behavioral data	After-school physical activity data
		Physical function and quality evaluation
		Medical index diagnosis
Sports competition and event information	Physical health diagnosis and evaluation	Mental state diagnosis
		Exercise prescription design
		Exercise prescription implementation
	Physical education curriculum intervention	Supervised exercise prescription evaluation feedback
Sports venue equipment resource management	Sports society club	Recommended course selection
		Course assessment
		Course evaluation
		Morning exercise program registration
		Morning exercise assessment

**Table 2:** Intuitive fuzzy number conversion between zones.

Language value	Interval intuitionistic fuzzy numbers
Very good (VG)	([3.8, 1.9], [0.05, 0.1])
Good (G)	([0.7, 2.8], [0.1, 0.2])
Generally good (MG)	([0.3, 0.7], [0.5, 8.3])
General (M)	([0.45, 0.55], [0.4, 0.45])
Average poor (MP)	([0.3, 0.4], [0.5, 4.6])
Poor (P)	([0.2, 6.3], [0.6, 0.7])
Very poor (VP)	([0.1, 0.2], [0.9, 0.8])

**Table 3:** Objective needs.

Projects of particular interest	Cannot or do not know whether it can achieve the purpose of promoting good health	No items of particular interest	Will accept recommended sports	Actively choose to participate in sports according to sports interests
24	46	39	24	54
57	40	45	39	31
47	49	35	45	38
44	54	32	23	20
23	40	32	25	52
44	25	58	26	55
37	49	48	57	46

## Data Availability

The data used to support the findings of this study are available from the corresponding author upon request.
